The article "Identification of XMRV Infection-Associated microRNAs in Four Cell Types in Culture" was retracted in 2013. Reasons: errors in the analysis; unreliable results or conclusions; concerns about the results or conclusions.

# Identification of XMRV Infection-Associated microRNAs in Four Cell Types in Culture

**DOI:** 10.1371/journal.pone.0032853

**Published:** 2012-03-16

**Authors:** Ketha V. K. Mohan, Krishnakumar Devadas, Shilpakala Sainath Rao, Indira Hewlett, Chintamani Atreya

**Affiliations:** 1 Section of Cell Biology, Laboratory of Cellular Hematology, Center for Biologics Evaluation and Research, Food and Drug Administration, Bethesda, Maryland, United States of America; 2 Laboratory of Molecular Virology, Center for Biologics Evaluation and Research, Food and Drug Administration, Bethesda, Maryland, United States of America; National Institute of Health, United States of America

## Abstract

**Introduction:**

XMRV is a gammaretrovirus that was thought to be associated with prostate cancer (PC) and chronic fatigue syndrome (CFS) in humans until recently. The virus is culturable in various cells of human origin like the lymphocytes, NK cells, neuronal cells, and prostate cell lines. MicroRNAs (miRNA), which regulate gene expression, were so far not identified in cells infected with XMRV in culture.

**Methods:**

Two prostate cell lines (LNCaP and DU145) and two primary cells, Peripheral Blood Lymphocytes [PBL] and Monocyte-derived Macrophages [MDM] were infected with XMRV. Total mRNA was extracted from mock- and virus-infected cells at 6, 24 and 48 hours post infection and evaluated for microRNA profile in a microarray.

**Results:**

MicroRNA expression profiles of XMRV-infected continuous prostate cancer cell lines differ from that of virus-infected primary cells (PBL and MDMs). miR-193a-3p and miRPlus-E1245 observed to be specific to XMRV infection in all 4 cell types. While miR-193a-3p levels were down regulated miRPlus-E1245 on the other hand exhibited varied expression profile between the 4 cell types.

**Discussion:**

The present study clearly demonstrates that cellular microRNAs are expressed during XMRV infection of human cells and this is the first report demonstrating the regulation of miR193a-3p and miRPlus-E1245 during XMRV infection in four different human cell types.

## Introduction

XMRV is a recently identified gammaretrovirus, closely related to xenotropic murine leukemia viruses (MLVs), that was initially detected in familial cases of prostate cancer tissue using a virus gene array [1]. XMRV was also detected in blood cells of patients with Chronic Fatigue Syndrome (CFS) and normal healthy controls [2], [3]. Subsequently, a number of additional studies have failed to confirm any association of XMRV with CFS or prostate cancer [4]–[11]. Indeed, recent reports suggest that XMRV likely originated as a laboratory contaminant in prostate xenografts serially passaged through nude mice by the recombination of endogenous MLVs. Though the XMRV is of murine origin, it is known to infect different human cell types like T and B lymphocytes, NK cells, prostate cancer cell lines, and neuronal cells [12]–[15]. Various detection methods like serology, cell culture, and nucleic-acid based assays have already been used for detecting XMRV infection [4], [12], [16]–[19]. However, use of microRNAs (miRNAs) as biomarkers of XMRV infection has not been reported so far.

The article "Identification of XMRV Infection-Associated microRNAs in Four Cell Types in Culture" was retracted in 2013. Reasons: errors in the analysis; unreliable results or conclusions; concerns about the results or conclusions.

MicroRNAs have known to play a critical role in the life cycle of retroviruses and a few oncogenic viruses such as reticuloendotheliosis virus strain T (REV-T), Epstein-Barr virus and Hepatitis C virus (HCV) wherein the viruses regulate host cells and viral replication through specific microRNAs [20]–[23]. MicroRNAs are a class of evolutionarily conserved, endogenous, small non-coding RNAs that regulate gene expression and play a role in diverse cellular processes, including proliferation, differentiation and cell death [24]. As an abundant class of regulatory molecules, there are hundreds of distinct miRNAs identified in the human genome to date and hundreds more predicted. A single miRNA can regulate expression of multiple genes, and expression of a single gene may be regulated by several distinct miRNAs, creating complicated regulatory networks. It is estimated that roughly 60% of human protein-coding genes are regulated by miRNAs [25]–[28].

In this study, we evaluated whether miRNAs are modulated by XMRV in cultured cells and if so, can they be identified to see whether a single or a set of miRNAs specific to the infection can be detected early that could serve as biomarker(s) of XMRV infection. Our results demonstrate that a) two miRNAs, miR-193a-3p and miRPlus-E1245 (a proprietary sequence of Exiqon Inc, Denmark and named as such to differentiate from miR-1245) were commonly regulated among all 4 cell types infected with XMRV used in the study, and b) while miR-193a-3p is down regulated, miRPlus-E1245 exhibited varied expression profile in the four cell types infected with XMRV.

## Materials and Methods

### Cell culture and isolation and culture of Peripheral Blood Lymphocytes (PBL)

LNCaP (ATCC, Manassas, VA) and DU145 cells (kind gift from Robert Silverman, Cleveland Clinic, Ohio to Indira Hewlett) were cultured in RPMI 1640 supplemented with 10% FBS, 2 mM glutamine, 100 units/ml of penicillin, and 100 units/ml streptomycin [29], [30]. PBMC were isolated from the peripheral blood of HIV seronegative donors (NIH Blood Bank) by Ficoll/Hypaque density gradient centrifugation. Monocytes were removed by adherence to the culture flasks and the remaining Peripheral Blood Lymphocytes (PBL) were stimulated with 2 µg/ml PHA for 3 days to activate T cells before infection. The PBL were cultured in RPMI 1640 supplemented with 10% FBS, 2 mM glutamine, 100 units/ml of penicillin, 100 units/ml of streptomycin, and 5 units/ml of human Interleukin-2 (Roche, NJ) until further use.

The article "Identification of XMRV Infection-Associated microRNAs in Four Cell Types in Culture" was retracted in 2013. Reasons: errors in the analysis; unreliable results or conclusions; concerns about the results or conclusions.

### Isolation and culture of Monocyte-derived Macrophages **(**MDMs**)**

Monocytes were isolated from PBMC of donors seronegative for HIV-1 and hepatitis B after leukopheresis and purified by countercurrent centrifugal elutriation [31]. Cell suspensions contained >95% monocytes by criteria of cell morphology on Wright-stained cytosmears, by granular peroxidase and by non-specific esterase. The cells were cultured for 5 days in DMEM supplemented with 10% FBS, 2 mM glutamine, 100 units/ml of penicillin, and 100 units/ml streptomycin and 1000 U/ml macrophage colony stimulation factor (M-CSF) before infection with XMRV. All cell culture reagents were tested by Limulus Lysate assay (Associates of Cape Cod, Cape Cod, MA) for endotoxin contamination and the levels were found to be <0.06 EU/ml.

### Infection with XMRV

Prostate cell lines LNCaP and DU145, Peripheral Blood Lymphocytes (PBL) and Primary monocyte-derived macrophages (MDM) were infected with 1×10^7^ XMRV copies/mL. After a three-hour exposure, virus particles were removed, and fresh medium was added and cultured at 37°C. Infected cells were isolated at the indicated times, washed twice in 1×PBS and stored at –80°C until further use.

### Cellular total mRNA extraction

Total RNA from the four cell types stored as above was extracted by using miRCURY™ RNA isolation kit as per the manufacturer's instructions (Exiqon, Denmark). The final volume of RNA extracted from each column was approximately 75–100 µl which was quantified by Nanovue® Plus spectrophotometer (GE Life Sciences, Piscataway, NJ). All the above experiments were conducted twice and RNAs extracted from duplicate experiments were analyzed for microRNA (miR) expression profile.

**Figure 1:** Quantitative-PCR analysis of XMRV infection. Total mRNA from (A) LNCaP, (B) DU145, (C) PBLs and (D) MDM cells either mock- or virus-treated were subjected to RT-PCR using the gag primers for detecting XMRV infection. GAPDH primers were used as endogenous controls. As evident, XMRV was able to infect all 4 cell types with substantial increase in infection by the 48 h time point.

### Quantitative RT-PCR

The endogenous human Glyceraldehyde 3-phosphate dehydrogenase (GAPDH) control real-time PCR primers and probes (TaqMan endogenous human GAPDH control, Cat# 4352934E) and the XMRV *gag* gene specific real-time PCR primers and probes were obtained from Applied Biosystems, Foster City, CA. Thermal cycling was performed for XMRV and GAPDH in triplicate on RNA samples in a Micro-Amp Optical 96-well reaction plate (Applied Biosystems, Foster City, CA). Briefly, an equal amount of total RNA was used to quantify XMRV levels using QuantiTect Probe RT-PCR kit (Qiagen Inc., Valencia, CA). Real-time PCR Master Mix (Quantitect Probe RT-PCR, Qiagen Inc., Valencia, CA) was added to the RNA, forward (CGAGAGGCAGCCATGAAGG) and reverse (CCCAGTTCCCGTAGTCTTTTGAG) *gag* primers, probe (6FAM-AGTTCTAGAAACCTCTACACTC-MGBNFQ) and primer for XMRV viral RNA first strand synthesis (reverse-transcription) (GAGATCTGTTTCGGTGTAATGGAAA) in a total volume of 25 µL. The mixture was incubated at 50°C for 2 min (for RNA, 20 min), at 95°C for 10 min, and then cycled at 95°C for 15 sec and 60°C for 60 sec 40 times, in an Applied Biosystems 7500 sequence detection system. XMRV levels were quantified using XMRV clone VP62-pcDNA3.1 (GenBank accession no. EF185282; obtained through NIH AIDS Research and Reference Reagent Program) as a standard. Each experimental sample was normalized relative to the GAPDH endogenous control and the relative amount of target gene quantified.

The article "Identification of XMRV Infection-Associated microRNAs in Four Cell Types in Culture" was retracted in 2013. Reasons: errors in the analysis; unreliable results or conclusions; concerns about the results or conclusions.

### Assessment of miRNA Quality and Array analysis

MicroRNA array services were contracted out to Exiqon Services, Denmark. The quality of the total RNA was verified by an Agilent 2100 Bioanalyzer profile. 1000 ng total RNA from sample and reference was labeled with Hy3™ and Hy5™ fluorescent label, respectively, using the miRCURY LNA™ microRNA Power Labeling Kit, Hy3™/Hy5™ (Exiqon, Denmark) following the procedure described by the manufacturer. The Hy3™-labeled samples and a Hy5™-labeled reference RNA sample were mixed pair-wise and hybridized to the miRCURY LNA™ microRNA Array (5th gen-hsa, mmu & rno) (Exiqon, Denmark), which contains capture probes targeting all miRNAs for human, mouse or rat registered in the miRBASE 16.0. The hybridization was performed according to the miRCURY LNA™ microRNA Array instruction manual using a Tecan HS 4800™ hybridization station (Tecan, Austria). After hybridization the microarray slides were scanned and stored in an ozone free environment (ozone level below 2.0 ppb) in order to prevent potential bleaching of the fluorescent dyes. The miRCURY™ LNA array microarray slides were scanned using the Agilent G2565BA Microarray Scanner System (Agilent Technologies, Inc., USA) and the image analysis was carried out using the ImaGene 9.0 software (BioDiscovery, Inc., USA). The quantified signals were background corrected (normal exposure with offset value 10) and normalized using the global LOWESS (LOcally WEighted Scatterplot Smoothing) regression algorithm [32].

The article "Identification of XMRV Infection-Associated microRNAs in Four Cell Types in Culture" was retracted in 2013. Reasons: errors in the analysis; unreliable results or conclusions; concerns about the results or conclusions.

**Figure 2:** Principal Component Analysis (PCA) Plot. The principal component analysis is performed on all samples and on all microRNAs with standard deviation over 1. The normalized log ratio values have been used for the analysis. Abbreviations: LM (LNCaP Mock); LV (LNCaP Virus-treated); DM (DU145 Mock); DV (DU145 Virus-treated); PM (PBL Mock); PV (PBL Virus-treated); and MM (MDM Mock); MV (MDM Virus-treated). The LNCaP and DU145 cell lines form tight cluster indicating minimal variation with regard to infection status and time. PBLs and MDMs are more spread suggesting variation due to both and time and infection status.

## Results

### Quantitative RT-PCR demonstrates XMRV infection in all 4 cell types studied

XMRV infection in the 4 cell types was determined by performing a quantitative RT-PCR (qPCR) on the total RNAs extracted at various time points. Endogenous GAPDH levels were used for normalizing the expression levels of the XMRV *gag* target gene. Results demonstrated that XMRV was able to infect all 4 cells types studied, very robustly in the prostate cell lines (LNCaP and DU145) and moderately in PBLs and MDMs (Fig. 1). A 3–10 fold increase in XMRV infection by 48 hours was evident among all 4 cell types (Fig. 1).

**Figure 3:** Heat map and unsupervised Hierarchical Clustering. The clustering is performed on all samples and on all microRNAs with standard deviation over 1. Each row represents one microRNA and each column represents one sample. The microRNA clustering tree is shown on the left. The color scale shown at the bottom illustrates the relative expression level of a microRNA across all samples: red color represents an expression level above mean, green color represents expression level lower than the mean.

### MicroRNA expression profiles of XMRV infected continuous cell lines differ from that of infected primary cells (PBL and MDMs)

Principal Component Analysis (PCA), a method used for reducing the dimension of large data sets and thereby useful to explore naturally arising sample classes/groups based on expression profile was performed. By including the microRNAs that have the largest variation across all samples (SD>1) an overview of how the samples cluster based on this variance is obtained. Based on this method, if the biological differences between various samples are pronounced, then this would become a primary component of the variation leading to segregation of samples in different regions of a PCA plot corresponding to their biology. As demonstrated in Fig. 2, it is observed that the overall miRNA expression profile in LNCaP and DU145 cell lines form a tight cluster suggesting minimal variation due to time and infection status of these two cell types, while the PBLs and MDM profiles are more spread, indicating the global miR levels being affected both due to time and infection status.

The article "Identification of XMRV Infection-Associated microRNAs in Four Cell Types in Culture" was retracted in 2013. Reasons: errors in the analysis; unreliable results or conclusions; concerns about the results or conclusions.

**Figure 4:** Identification of top 25 commonly regulated microRNAs in the four cell types tested. As seen in this venn diagram two miRs are commonly regulated in all four cell types. While 6 miRs were commonly regulated in 3 of the 4 cell types tested, 11 miRs were found to be common in at least 2 of the 4 cell types. Cell-type specific miR regulation was found to be 11 miRs each for PBL and DU145 cell lines and 16 miRs each were regulated in LNCaP and MDM cells.

### Heat map analysis and unsupervised hierarchical clustering

MicroRNA expression profiles from four different XMRV-infected cell types at 3 different time points were plotted on a heat map. As observed in Fig. 3, the heat map diagram depicts results of the two-way hierarchical clustering of microRNAs and samples. Each row representing one miRNA and each column representing one sample confirms the variation in miRNA expression profile between the continuous prostate cancer cell lines (LNCaP and DU145) and the PBLs and MDMs. A more distinct pattern of demarcation in miRNA profiles between these two set of cell types is observed in the region of the heat map depicting miR-1275 to miR-765 (Fig. 3). The microRNA clustering tree is shown on left of the figure.

**Figure 5:** Tabular representation of top 25 most differentially expressed miRs in the 4 cell types D-DU145; L-LNCaP; P-PBL, and M-MDMs). (Yellow represents miRNAs present in all 4 lists (hsa-miR-193a-3p and hsa-miRPlus-E1245), blue represents miRNA present in 3 out of 4 lists and dark-red represents miRNAs present in 2 out of 4 lists.

### miR-193a-3p and miRPlus-E1245 are specific to XMRV infection in all 4 cell types

The main objective of the current study was to identify common miRNAs that are uniformly regulated in all 4 cells types due to XMRV infection and hence an overall comparative analysis was performed. While comparing the two sample groups (mock versus infected) using a paired t-test, no microRNA was found to be differentially expressed using a cut-off of p-value<0.05. Since the experiment involved 4 cell lines that behave differently, with two treatments (mock- and virus-treated) and 3 time-points (6 h, 24 h and 48 h), a more logical approach was adopted to simply look into the differences between the two treatments over the three time-points, by subtracting the control (mock) from the virus treatment. Subsequently, the most differentially expressed genes between the 3 time points (6 h to 24 h and 48 h) was estimated. As represented in a venn diagram (Fig. 4) a total of 72 differentially expressed miRs were observed between the 4 four cell types. Among these, 2 miRs were common in all 4 cell types, while 6 miRs were found to be common in 3 of the 4 cell types and 11 miRs were common in at least 2 of the 4 cell types.

The article "Identification of XMRV Infection-Associated microRNAs in Four Cell Types in Culture" was retracted in 2013. Reasons: errors in the analysis; unreliable results or conclusions; concerns about the results or conclusions.

**Figure 6:** Differential expression of miR-193a-3p and miRPlus-E1245. By subtracting the miR expression values from the virus-infected and mock-infected (M-V) and further subtracting the values between the time points (▵T6▵T24 and ▵T6-▵T48) an expression profile was generated for the two miRs as mentioned above. It can be observed that miR-193a-3p is down regulated over time due to virus infection in all 4 cell types, whereas miRPlus-E1245 exhibits varied levels of expression profile between the 4 cell types.

Further analysis of the top 25 differentially expressed miRs between the 4 cell types revealed that the two miRNAs common to all 4 cell types were miR-193a-3p and miRPlus-E1245 (Fig. 5). The miRPlus-E1245 is a recently discovered miRNA and proprietary sequence of Exiqon Inc, Denmark and named as such to differentiate it from miR-1245. The sequence is not yet annotated and hence not been submitted to the miRNA database yet. More significantly, though the miRPlus-E1245 levels were in the top 25 list in one experiment and moderately regulated in the second experiment, the miR-193a-3p expression profile was among the top 25 list in both the microarray experiments. The reason for the observed differences in the relative abundance of the differentially expressed miRNAs could be due to donor-to-donor variations. MicroRNAs that were common in 3 of the 4 cell types were miR-15a, miR-19a, miR-29b, miR-32, miR-33a, and miR-101. Eleven microRNAs that were differentially expressed and common in 2 of the 4 cell types were found to be miR-17, miR-21, miR-29c, miR-141, miR-142-3p, miR-215, miR-494, miRPlus-E1072, miRPlus-E1192, miR-1248, and miR-1973 (Fig. 5).

### miR-193a-3p is down regulated and miRPlus-E1245 exhibits varied expression profile

Following the identification of 2 miRs (miR-193a-3p and miRPlus-E1245) that were specific to all 4 cell types infected with XMRV, it was logical to deduce the expression profile of these two miRNAs in all 4 cell types over time in virus-infected cells. By subtracting the miRNA expression values from the virus-infected and mock-infected (M-V) and further subtracting the values thus generated between the time points (▵T6-▵T24 and ▵T6-▵T48), an expression profile was generated for the two miRNAs as mentioned above. It can be observed in figure 5 that miR-193a-3p is down regulated over time due to the virus infection in all 4 cell types. The miRPlus-E1245 however exhibits varied levels of expression profile between the 4 cell types with up regulation in MDM and PBL cell types and down regulation in LNCaP and DU145 cell types (Fig. 6).

The article "Identification of XMRV Infection-Associated microRNAs in Four Cell Types in Culture" was retracted in 2013. Reasons: errors in the analysis; unreliable results or conclusions; concerns about the results or conclusions.

**Table 1:** Target prediction for miR-193a-3p using 3 different programs.

S.No	Gene description	Gene symbol	miRDB	TargetScan	microRNA.org
1	SON DNA binding domain	SON	+	+	+
2	Friend Leukemia virus Integration 1	FLI1	+	+	
3	Abl Interactor 2	ABI2	+	+	
4	v-erb-erythroblastic leukemia viral oncogene homolog 4 (avian)	ERBB4	+	+	
5	Solute carrier family 10 (Na/bile acid cotransporter family), member 6	SLC10A6		+	+
6	FH2 domain containing 1	FHDC1		+	+

Top 10 genes commonly picked by at least two different prediction programs are indicated.

## Discussion

The discovery of XMRV and its potential association with PC and CFS aroused considerable excitement and promise within the research and clinical community regarding a possible infectious etiology for at least some cases of these disease or conditions. [2], [3], [33]. However, recent research findings have not supported any association between the virus and CFS or prostate cancer [7], [9], [10], [34]–[37]. In fact, the virus itself may have originated as a result of recombination in a laboratory setting [38], [39]. Specifically, it has been postulated that XMRV originated as a result of recombination between two MLV proviruses in laboratory mice [40]. These findings appear to raise doubts about the significance and involvement of XMRV in any human disease or condition [38]–[41]. Nonetheless, because at least some studies have demonstrated that XMRV is a culturable virus and that it can readily infect cells of human origin [12]–[15], additional research efforts will help to further our understanding of XMRV pathogenesis and provide insights into the modes of transmission involved in XMRV infection. It also remains to be seen whether XMRV demonstrates potential to be transmitted across species [12], [37], [41].

The present study further emphasizes that XMRV can infect human prostate and hematopoietic cells and the study clearly demonstrates that microRNAs are regulated during XMRV infection of these culturable human cells. In fact, the qPCR results indicate that while all the 4 cell types were susceptible to XMRV infection with significant increase in viral titers by 48 h time point it was evident that there was a distinct difference in infection levels between the 4 cell types (Fig. 1). The prostate cell lines (LNCaP and DU145) supported robust XMRV infection, while the PBLs and MDMs were moderately infected. It is interesting to note that the variability in infection status of the 4 cell types may potentially be dependent on individual APOBEC levels in each cell type [42]. It has been shown earlier that XMRV is resistant to human APOBEC 3G (hA3G) and that the levels of hA3G are down-regulated by XMRV in LNCaP and DU145 cells thereby supporting efficient viral infection in these cell types [42], [43]. The hA3G is down regulated by the human immunodeficiency virus-1 (HIV-1) *vif* protein during infection. However, since XMRV lacks *vif*, an alternate mechanism of hA3G down regulation has been suggested [43]. PBMCs on the other hand, seemingly possess significantly higher levels of h3AG and hence are relatively resistant to XMRV infection [42].

The article "Identification of XMRV Infection-Associated microRNAs in Four Cell Types in Culture" was retracted in 2013. Reasons: errors in the analysis; unreliable results or conclusions; concerns about the results or conclusions.

The two microRNAs (miR-193a-3p and miRPlus-E1245) are moderately regulated in the four cell types. However, it is interesting to note that within the four cell types, miR-193a-3p is down regulated over time, while miRPlus-E1245 however exhibited varied levels of expression profile between the 4 cell types: up regulation in MDMs and PBL cell types and down regulation in LNCaP and DU156 cell types. Since the miRPlus-E1245 has not been annotated and not submitted in the miRNA database yet by its discoverer, the Exiqon Inc., Denmark, it is not feasible at this time to identify its potential targets. Therefore, we only analyzed the miR-193a-3p for its tentative mRNA targets by 3 different online programs as indicated in Table 1. Target Prediction by miRDB, TargetScan and microRNA.org programs revealed that out of the top 10 mRNA targets that were identified individually by these 3 different softwares, 1 target mRNA was picked by all three programs and 5 mRNA targets were commonly flagged at least by two different programs. Of the six predicted mRNA targets for miR-193a-3p, five mRNA targets were related to tumorogenesis or suppression. Interestingly 3 mRNA targets, namely SON DNA binding domain (SON), Friend Leukemia Virus Integration 1 (FLI1) and v-erb-erythroblastic leukemia viral oncogene homolog 4 (ERBB4) have been implicated with virus/virus infections. Of the 3, the FLI1 protein (or its homolog) may have a potential role in XMRV infection as this protein has already been implicated in Friend Leukemia Virus which also is a retrovirus causing tumorigenesis [44], [45]. The FLI1 is a protein responsible for the integration of the viral gene into the host DNA thereby leading to carcinogenesis [44], [45]. The human genome was recently analyzed for potential XMRV genome integration sites and results revealed that the virus had integration sites in at least 11 of the 23 chromosomes [46]. Hence it is to be seen whether this particular host mRNA target is being modulated by miR-193a-3p during XMRV infection. Of the other two, while the SON protein binds to hepatitis B virus (HBV) DNA and exhibits sequence similarity to other oncoproteins, the ERBB4 protein affects mitogenesis and cell differentiation and furthermore it is known that mutations within this gene are associated with cancer [47]–[49].

The article "Identification of XMRV Infection-Associated microRNAs in Four Cell Types in Culture" was retracted in 2013. Reasons: errors in the analysis; unreliable results or conclusions; concerns about the results or conclusions.

More pertinently, while the qPCR results revealed robust infection in two cell types (LNCaP and DU145 cells) and moderate infection in the other two tested cell types (PBLs and MDMs), what is common to all 4 cell types is the regulation of the two miRNAs (miR-193a-3p and miRPlus-E1245) during XMRV infection regardless of the level of infectivity, virus titer or dose of the infection. This is the first report indicating the expression and regulation of miRs during XMRV infection of human cells. It remains to be seen whether the same set of miRNAs are up regulated during infection of murine cells or cell lines.

The current findings reported here certainly demonstrate that XMRV infection modulates miRNAs in the host cells as is the case with many other viruses that are pathogenic to humans [20]–[23]. In human retroviruses such as HIV-1 and HTLV-1, the role of microRNAs has already been demonstrated [50]–[54]. Many of these exquisite studies have clearly shown how certain miRs up regulate or down regulate certain host genes/proteins to promote viral infection or disease pathogenesis [50]–[52], [54], [55]. In fact, it is now known that HIV-1 and other viruses themselves code for microRNAs, which play a critical regulatory role during virus infection [50], [56]. Our studies also demonstrate that miRNA profiles are different in XMRV-infected prostate cancer cell lines compared to primary hematopoietic cells, suggesting that miRNAs could play a role in XMRV infection, and serve as markers of XMRV infection in cultured cells.
